# Random Forest Algorithm Based on Speech for Early Identification of Parkinson's Disease

**DOI:** 10.1155/2022/3287068

**Published:** 2022-05-09

**Authors:** Ping Fan

**Affiliations:** School of Chinese Language and Literature, Nanjing Normal University, Nanjing, China

## Abstract

To investigate the effectiveness of identifying patients with Parkinson's disease (PD) from speech signals, various acoustic parameters including prosodic and segmental features are extracted from speech and then the random forest classification (RF) algorithm based on these acoustic parameters is applied to diagnose early-stage PD patients. To validate the proposed method of RF algorithm in early-stage PD identification, this study compares the accuracy rate of RF with that of neurologists' judgments based on auditory test outcomes, and the results clearly show the superiority of the proposed method over its rival. Random forest algorithm based on speech can improve the accuracy of patients' identification, which provides an efficient auxiliary method in the early diagnosis of PD patients.

## 1. Introduction

Parkinson's disease (PD) is a progressive neurodegenerative disease with ambiguous etiology. Although the exact reason is still unknown, the riskiest factor of PD is age, which causes the prevalence rate of PD to increase with the increase of age. The main pathological changes in patients with PD are the death and loss of dopaminergic neurons in the substantia nigra pars compacta which is irreversible. It means that patients with PD will never be cured, but anti-Parkinson's medication or deep brain stimulation surgery can slow down the progression of the disease [1]. So, early detection, early intervention, and early treatment of PD patients are essential to alleviate their pain and the burden of their families.

Patients with PD are usually diagnosed based on clinical symptoms (e.g., rest tremor, rigidity, and bradykinesia). In addition to traditional clinical symptoms, neuroimaging, genetic, and biochemical studies are applied for early detection of PD, whereas no reliable biomarkers can be used as the only valid criterion. Consequently, patients that are underdiagnosed and misdiagnosed are common [2]. A single biomarker is insufficient for the PD diagnosis, and a variety of methods need to be combined.

Speech characteristics that can serve as a novel clinical biomarker for PD diagnosis have been noticed by researchers. A longitudinal study has shown that the disturbance of speech acoustic parameters in Parkinson's disease (atypical range and variance of the fundamental frequency) occurs approximately 5 years before the onset of clinical symptoms [3]. Other related studies mainly focus on the speech differences between PD and healthy speakers which manifest in multiple speech subsystems, including phonation, articulation, and prosody, which can be used to distinguish PD patients from healthy adults [4].

Although speech disorder may be an early sign of PD, it is usually ignored by patients themselves and their caregivers [5, 6]. So, investigating the speech characteristics in PD patients, especially for patients in their early stages, is vital to early diagnosis of PD patients. Nevertheless, few studies have reported the contributions of speech features in the identification of PD patients.

## 2. Literature Review

As stated by previous studies, changes in prosodic and segmental speech features of speech (e.g., speech rate and articulatory deficits) are among the early symptoms in PD patients, whereas the difference in phonation features of Parkinsonian and healthy speech is not significant [5,7]. So, prosodic and segmental features of PD speech are reviewed in the current study.

Less variability of fundamental frequency (F0) and narrower F0 range which are in close relation with monopitch or monotone is the most prominent feature of PD speech [8]. Previous studies have confirmed that F0 disorders in PD speakers exist not only in the prodromal stage but also in the later stage of the disease [7]. Rusz et al. [9] reported that F0 variability is one of the most reliable acoustic indicators of Parkinson's disease. Studies targeting the relationship between acoustic features of PD speech and their motor symptoms show a significant negative correlation between F0 variability of parkinsonian speech and disease progression, with an explanation that the movement of vocal folds in PD patients is sensitive to reflect disease progression [10].

Deficits in speech timing are also observed in early PD speakers [11, 12]. Speech rate is affected by Parkinson's disease [13]. Compared to healthy speakers, PD patients speak at a faster or slower rate, showing a great individual variability [14]. Although speech rate has been used to study the pathological change in PD speech, its reliability to differentiate speakers with PD from healthy speakers remains uncertain. Rhythmic metrics play an important role in distinguishing pathological speech from normal speech. Liss et al. [15] stated for the first time that a set of rhythmic metrics (e.g., standard deviation of consonantal durations and proportion of vocalic durations) can be used to distinguish speakers with dysarthria from healthy individuals. In particular, Lowit et al. [12] found the proportion of vocalic durations in speech is a robust indicator of PD.

Studies of motor speech disorders have been focused on vowel production to investigate articulation impairments, and thus articulation deficits have been extensively studied in PD speakers. Vowel articulation impairment is considered an important marker for early-stage PD speakers [16, 17]. Various indices such as the ratio between the second formant of the vowels /i/ and /u/ (*F*2_i_/*F*2_u_), vowel space area (VSA), and vowel articulation index (VAI) are used to characterize vowel articulation in previous studies; however, these studies show inconsistent results. Several studies show that VSA is less reliable than VAI in identifying PD speakers suffering from mild dysarthria [17–19], while other studies conclude that both VAI and VSA can identify articulation disorders of PD speakers [16].

Inconsistent results are also observed for stops in the PD speech. Longer voice onset times (VOTs) of consonants have been observed in PD speech [20, 21]. On the other hand, Ackermann and Ziegler [22] and Kim [23] found that stops have shorter VOTs in PD speech. Moreover, a recent study has found that there is no significant difference in VOT between speakers with PD and healthy individuals [24].

Although acoustic differences in speech between individuals with PD and healthy speakers are well documented, little is known about which acoustic features are the most important in distinguishing PD patients, in particular early-stage ones, from healthy adults. In contrast, neurologists usually use clinical scales such as the United Parkinson's Disease Rating Scale [25], which however is subjective and may mislead their judgments of PD patients.

Therefore, this study focuses on two questions. First, which metrics are the most important in differentiating PD from healthy speakers? Second, is automatic classification more advantageous in identifying PD patients than auditory perception? To investigate these two questions, the machine learning algorithm based on both prosodic and segmental features of speech is used to explore the relative contributions of acoustic features and the accuracy rate of early-stage PD identification. Then, neurologists are recruited to judge whether the speaker is a PD patient or not after they hear the reading speech. The accuracy rate is compared with that of automatic classification.

## 3. Methods

To solve the two problems raised above, this study recruited PD patients in early stages and recorded their reading speech in quiet rooms (noise < 50 dB). Based on the reading speech, several acoustic metrics of speech are extracted. All speech data are divided into two sets, i.e., training set and testing set. Using random forest classification, we explored the accuracy rate of classification of early-stage PD patients and the relative contributions of these acoustic metrics to the classification. The framework of this study is shown in Figure 1.

### 3.1. Participants and Materials

To minimize the effects of dialects and special speaking styles on acoustic results, speakers who spoke with an accent or spoke in an unusual way were screened out [26]. So, thirty-six individuals with idiopathic PD (19 men and 17 women) aged 52 to 78 years (mean = 63.55, SD = 9.46) were recruited as the PD group. The Hoehn and Yahr score of PD was between 1 and 2.5, and the disease duration was less than 5 years, which meant that all patients were in the early stage of PD [27]. None of the patients had suffered from other diseases or had undergone deep brain stimulation surgery. All participants were native Mandarin speakers and scored at least 24 on the Mini-Mental State Exam.

Speech task is an important factor in voice disorder investigation [11, 28]. According to previous studies, passage reading is the optimum task to explore PD speech compared with sustained vowels and fast syllable repetition [21, 29], so passage reading is used in the current study. Before speech recording, the participants were instructed to read silently the passage *The North Wind and the Sun,* which consisted of 169 syllables in Mandarin. Then, all participants read the passage in a quiet room and speech was recorded using a Zoom H4n portable recorder at a sampling rate of 44100 Hz. The English translation of this passage is shown below.

The North Wind and the Sun were disputing which was the strongest, when a traveller came along wrapped in a warm cloak. They agreed that the one who first succeeded in making the traveller take his cloak off should be considered stronger than the other. Then, the North Wind blew as hard as he could, but the more he blew, the more closely did the traveller fold his cloak around him, and at last the North Wind gave up the attempt. Then, the Sun shined out warmly, and immediately the traveller took off his cloak, and so the North Wind was obliged to confess that the Sun was the strongest of the two.

To avoid the influence of anti-Parkinson medication on speech production, speakers of PD stopped taking medication and were in a fasting state for at least 12 hours before the speech recording.

### 3.2. Acoustic Measures

Acoustic analysis was conducted on two aspects of acoustic measures. One aspect was the prosodic feature (fundamental frequency parameters, speech rate, and rhythm), and the other was the segmental feature (formants of vowels and voice onset time of stops). Details of the 13 acoustic measures are described below.

The measures of the fundamental frequency (*F*0) were extracted from the Praat software. The autocorrelation algorithm in Praat generated F0 tracks for every speech sample, and then gross *F*0 errors were manually corrected according to the waveform and spectrogram. Five *F*0 parameters were calculated from the *F*0 tracks, namely, the minimum (*F*0min), maximum (*F*0max), mean (*F*0mean), range (difference between *F*0min and *F*0max, *F*0range), and standard deviation of *F*0 (F0std). All *F*0 values were converted from Hz to semitones (St) with 50 Hz as the reference frequency. The formula is as follows (fr is the *F*0 value in Hz).

(1) $$\begin{array}{c} \text{St}=12\times \;\log_{2}\left(\frac{\text{fr}}{50}\right)\;. \end{array}$$

Both speech rate and articulation rate were calculated. Speech rate was defined as the total number of syllables divided by the total speech duration, and articulation rate was defined as the total syllables divided by the articulation duration. Pauses longer than 200 ms were marked and excluded from the measurement of articulation rate [30].

(2) $$\begin{array}{c} \text{Speech rate}=\frac{\text{the numbers of syllables}}{\text{total speech duration}},\\ \text{articulation rate}=\frac{\text{the number of syllables}}{\text{total speech duration}-\text{pause duration}}. \end{array}$$

Among the rhythmic parameters commonly used to distinguish different types of language [31], proportion of vowel vocalic durations in speech (%*V*) was reported to be effective in identifying speakers with brain injury and Parkinson's disease as reported [12, 32], so %*V* was investigated as a rhythmic measure in this research.

(3) $$\begin{array}{c} \%V=\frac{\text{vocalic duration}}{\text{total speech duration}}\times 100\%\;. \end{array}$$

Vowel articulation was measured by the ratio of the second formants of the vowels /i/ and /u/ (*F*2i/*F*2u), and the triangular vowel space area (tVSA) and the vowel articulation index (VAI) were based on the corner vowels /a, *i*, u/ in the speech sample. The middle 60% interval of the whole vowel was extracted from the monosyllables containing these three vowels to obtain the stable values of the first and second formants (*F*1 and *F*2) of these three vowels. tVSA with unit Hz^2^ has been widely used to measure the distribution of vowels, and VAI has been associated with the concentration or dispersion of vowels. The more concentrated the vowels, the smaller the VAI (the minimum of VAI is 0.5). The formulas for tVSA and VAI are as follows [17]:

(4) $$\begin{array}{c} \text{tVSA}=\text{ABS}\left\{\frac{\left[F1\left[i\right]\times \left(F2\left[a\right]-F2\left[u\right]\right)+F1\left[a\right]\times \left(F2\left[u\right]-F2\left[i\right]\right)+F1\left[u\right]\times \left(F2\left[i\right]-F2\left[a\right]\right)\right]}{2}\right\},\\ \text{VAI}=\frac{F2\left[i\right]+F1\left[a\right]}{F1\left[i\right]+F1\left[u\right]+F2\left[u\right]+F2\left[a\right]}. \end{array}$$

Voice onset time (VOT) of stops reflects the precise time coordination between the movements of the supra laryngeal articulators (such as lips and tongue) and the vocal folds. In this study, the VOTs of the post-pausal stops /*p*, *p*^*h*^, *t*, *t*^*h*^, *k*/ were compared between the two groups. Considering that speech rate has a direct impact on VOT, a normalized parameter, VOT ratio, was used in this study [24].

(5) $$\begin{array}{c} \text{VOT ratio}=\frac{\text{VOT}}{\text{syllable duration}}\times 100\%. \end{array}$$

Because VOT is longer for aspirated stops than for unaspirated stops in Mandarin, the VOT ratios of post-pausal stops were calculated for aspirated /*p*^*h*^, *t*^*h*^/ and unaspirated /*p*, *t*, *k*/ (hence VOT ratio_un and VOT ratio_as), respectively. All the 13 acoustic measures are summarized in Table 1.

### 3.3. Random Forest Classification

Based on all these acoustic parameters, a random forest classification in R [33] was used to investigate the contribution of these acoustic parameters to the classification of PD individuals and healthy controls.

First, the minimum value of the mean error rate of the model was calculated based on out-of-bag (OOB) data, and the optimal number of variables of the binary tree in the node “mtry” was set to 3 in the package randomForest. Since the model error tends to converge when the number of decision trees approaches 500, the optimal number of decision trees nTree was set to 500. Among the experimental data, 70% were randomly selected as the training set and the remaining 30% were selected as the test set. Finally, the accuracy, sensitivity, and specificity were calculated.

### 3.4. Auditory Perception Test

To compare the effectiveness of acoustic classification and the auditory judgment by neurologists, an auditory perception test was performed.

An utterance of the following sentence for about 10 seconds: “They agreed that the one who first succeeded in making the traveller take his cloak off should be considered stronger than the other,” was selected from speech recording from each participant, so that 36 stimuli were collected as auditory stimuli. Five neurologists who had been working in the department of neurology for at least 2 years were recruited in the auditory perception test. All five listeners had rich clinical experience in the assessment of patients with PD, but they were unaware of the purpose of the study.

After the intensity was normalized to 70 dB using the Praat software, all 36 speech stimuli were played back in a random order to the listeners through earphones in a quiet room. The following prompt was displayed on the computer screen: “Please judge from the speech you heard whether the speaker is a patient with PD.” Then, after each speech stimulus was played back, two options appeared on the computer screen: “PD patients” and “healthy persons.” Listeners clicked the mouse to complete the forced choice.

## 4. Results

### 4.1. Results of Random Forest Classification

The results based on 13 acoustic measures showed that the classification accuracy of the random forest algorithm was 75.6%, and the sensitivity and specificity were 66.7% and 84.6%, respectively.

Figure 2 shows the importance of all 13 acoustic measures in distinguishing PD patients from healthy controls. The most important measures in identifying speakers with early PD were F0std, F2i/F2u, F0 range, and VAI.

### 4.2. Results of Auditory Perception Test

The perceptual accuracy of five neurologists ranged from 61.1% to 68.1%, with a mean accuracy of 64.2%, which was lower than the accuracy of random forest classification (75.6%).

## 5. Discussion

Speech disorders have been well documented in previous studies, whereas the current study focuses on the contributions of prosodic and segmental features of early PD speakers and the superiority of acoustic classification using the random forest algorithm to clinical auditory judgments.

The random forest classification based on 13 acoustic measures including both prosodic and segmental features showed that the most important measures in identifying early PD speakers were F0std, F2i/F2u, F0 range, and VAI. Among these 4 acoustic measures, F0std and F0 range were prosodic features while F2i/F2u and VAI were segmental features. The smaller F0 range and F0 variability (F0std) in the early-stage PD speakers suggested their less expressive pitch variation, consequently resulting in monotone as previous studies reported [3, 9]. Although previous studies reported that either F0 parameters or vowel articulation played roles in distinguishing PD from healthy speakers [9, 17], the current study further showed that both F0 and vowel articulation were important in identifying individuals with early PD.

The identification accuracy of speakers with early-stage PD was 75.6%, which was higher than that of auditory assessment by neurologists. Therefore, this objective algorithm could be an effective auxiliary method for neurologists to identify speech disorders in early-stage patients with PD that were not easily perceptible.

It should be noted that the accuracy of identifying speakers with early PD based only on acoustic measures was 75.6%, still far away from being perfect. There were two possible reasons. First, not all speakers with early PD had speech disorders. Second, in addition to these acoustic measures we investigated here, some other parameters may also play roles in distinguishing early PD patients from healthy individuals. Therefore, our future study will explore more acoustic metrics and conduct multiple tasks, e.g., monologue and dialogue, to make a better identification of early-stage PD.

## 6. Conclusion

Random forest classification algorithm based on acoustic measures, especially fundamental frequency and vowel articulation, can be an auxiliary method to identify early-stage PD. There are diverse early biomarkers of PD such as clinical symptoms and neuroimages. However, the value of a single biomarker for early diagnosis is limited, and a variety of methods can be combined to improve the accuracy of diagnosis. The result of our research shows that a classification model based on speech acoustic parameters can provide a more economical, convenient, and effective way for early diagnosis, accurate assessment, and remote monitoring of PD patients. Nevertheless, acoustic parameters extracted from reading speech in this study are not yet comprehensive, and more acoustic features and multiple speech tasks should be considered in future studies.

## Figures and Tables

**Figure 1:** Framework of this study.

**Figure 2:** Importance of acoustic measures.

**Table 1:** Acoustic measures extracted from speech.

Acoustic measure	Type of feature
*F*0min (St)	Prosody
*F*0max (St)	
*F*0mean (St)	
*F*0range (St)	
*F*0std (St)	
Articulation rate (syl/s)	
Speech rate (syl/s)	
%*V*	

*F*2i/*F*2u	Segments
tVSA (kHz^2^)	
VAI	
VOT ratio_un	
VOT ratio_as	

## Data Availability

The data used to support the findings of this study are available from the corresponding author upon request.
